The article "Deep Learning Neural Network Prediction System Enhanced with Best Window Size in Sliding Window Algorithm for Predicting Domestic Power Consumption in a Residential Building" was published in 2022. Journal: Comput Intell Neurosci.

# Deep Learning Neural Network Prediction System Enhanced with Best Window Size in Sliding Window Algorithm for Predicting Domestic Power Consumption in a Residential Building

**DOI:** 10.1155/2022/7216959

**Published:** 2022-03-02

**Authors:** Dimpal Tomar, Pradeep Tomar, Arpit Bhardwaj, G. R. Sinha

**Affiliations:** ^1^Gautam Buddha University, Greater Noida, UP, India; ^2^BML Munjal University, Gurugram, Haryana, India; ^3^MIIT Mandalay, Mandalay, Myanmar

## Abstract

Buildings are considered to be one of the world's largest consumers of energy. The productive utilization of energy will spare the accessible energy assets for the following ages. In this paper, we analyze and predict the domestic electric power consumption of a single residential building, implementing deep learning approach (LSTM and CNN). In these models, a novel feature is proposed, the “best N window size” that will focus on identifying the reliable time period in the past data, which yields an optimal prediction model for domestic energy consumption known as deep learning recurrent neural network prediction system with improved sliding window algorithm. The proposed prediction system is tuned to achieve high accuracy based on various hyperparameters. This work performs a comparative study of different variations of the deep learning model and records the best Root Mean Square Error value compared to other learning models for the benchmark energy consumption dataset.

## 1. Introduction

Today's modern world faces steady acceleration in the development of technology, population, and economic growth, which dramatically increases energy consumption. As per the International Energy Agency (IEA) report, more than 30% of the global energy is consumed in buildings, and nearly one-third of carbon dioxide (CO_2_) emitted by the building accounts for a significant part of the total CO_2_ emissions [1]. Hence, buildings are the world's prime consumers of energy, and broadly, in residential sectors, heating and cooling systems consume energy, accounting for more than one-fifth of the total [2]. Though being a good consumer of energy, buildings are also connected with a significant proportion of energy waste as well [3], and this dissipated form of energy shows an alarming situation to sustainability. Such frightening circumstances address the concerns of growing energy demand, development of urbanization, and pollutant emissions, the increasing need of new smart sustainable energy resources. Hence, it is necessary to emerge with solutions that deal with building energy efficiently as it is extremely crucial. With this pattern, accurate predictions of future electric power consumption have become a fundamental advance in the computerized administration of power systems.

The article "Deep Learning Neural Network Prediction System Enhanced with Best Window Size in Sliding Window Algorithm for Predicting Domestic Power Consumption in a Residential Building" was published in 2022. Journal: Comput Intell Neurosci.

We can abate the further rise in the above-mentioned primary issues, namely, pollutant emissions (e.g., CO_2_) and energy consumption in buildings, only by promoting energy-saving designs for buildings during the design phase [4]. To accomplish smart and sustainable designs for energy efficiency, a focus has been derived towards the integration of buildings and smart technology for modeling and forecasting energy consumption. A smart environment is composed of “networks of sensors” that produce substantial amounts of energy data [5], for instance, the smart grid, the next level of the future power grid that dynamically deals with the generation and distribution of energy; therefore, at aggregate as well as modular level, smart, intelligent, and reliable decisions should be made endlessly in the grid with flexibility [6]. However, to achieve the reliability and efficiency of the grid, it is important to predict the future energy demand. In addition to that, smart meters are also quite promising in understanding the behavior of energy consumption with better clarity to the consumers as they do not save energy by themselves and are capable of sending precise readings to the power suppliers for customer billing. However, during the past decades, various countries like the United States of America (USA), China, and Europe have been working on energy efficiency by conducting programs of deploying smart meters at a large scale [7–10]. This smart technology will benefit in lowering electricity bills and optimizing power consumption, which will play a significant role in the development of sustainable smart cities and societies. But, we should take into account that innovation and technology all alone will not be sufficient to change how individuals devour energy, yet it gives the intention to utilize energy in a purposeful and cognizant manner. Furthermore, resident's behavior and households count are the secondary factors having a substantial influence on the energy efficiency profile of domestic buildings. Particularly, the occupancy of various household appliances is primarily responsible for obtaining the household electric power consumption. Beckel, Sadamori and Staake [11] reveal characteristics of the households, number of occupants, and appliances using energy-related data generated from smart meters. Haldi and Robinson [12] tried to predict the impact of occupant's behavior and their presence on the energy demand in buildings.

Artificial intelligence (AI) techniques have been applied in a wide range of disciplines and attracted the attention of researchers or scientists. AI models perform powerful data modeling by simulating the obtained information and adapt to changes in historical data to infer new facts [13]. Various qualitative works have recognized that AI techniques like statistical and learning-based modeling are ample skillful to apprehend nonlinear and tricky relationships that yield extremely good accuracy estimates from the historical energy-related data of buildings [13–15]. These AI models are quite promising for the prediction of domestic energy consumption in residential buildings accurately. However, it widely depends upon the researcher's requirement and their work on how to derive these AI models. Also, the success of AI techniques usually relies upon “data representation.” Out of them, deep learning aspires to form a combination of various nonlinear transformations and helpful interpretation in a more abstractive way and ultimately achieve more benefit [16]. Hence, the deep learning approach has been vigorously considered in different application areas such as image and video recognition [17–20], speech recognition [21, 22], and natural language processing [23, 24].

The article "Deep Learning Neural Network Prediction System Enhanced with Best Window Size in Sliding Window Algorithm for Predicting Domestic Power Consumption in a Residential Building" was published in 2022. Journal: Comput Intell Neurosci.

The deep recurrent neural networks are powerful tools dealing with the long sequence modeling in various domains of time series like energy demand and usage prediction. This work chooses Long Short-Term Memory (LSTM) and Convolution Neural Network (CNN) with an enhanced sliding window algorithm for predicting domestic energy consumption. The advantages of this enhanced deep learning model include (1) capturing the nonlinear correlation over multivariable energy data composed of exogenous and target variables, (2) modeling the temporal information into separable spaces for energy predictions, (3) identifying the best “N” window size, that is, the number of days considerable in the past that yields the optimal models followed by the best N window size graph for both the deep learning models, and (4) hyperparameter tuning of the models for more accurate predictions.

### 1.1. Related Work

Several studies have been devoted to predicting energy consumption at an industrial and residential level. Analyzing energy performance in buildings, which has been the subject of many researchers, is categorized into two modeling approaches: traditional statistical approach and machine learning approach.  Table 1 presents the summary of researches conducted on energy consumption in buildings and their proposed method based on two categories, namely, conventional statistical methods and traditional machine learning modeling.

#### 1.1.1. Conventional Statistical Methods

Conventional statistical methods are popular and classical modeling techniques that have been widely used to solve forecasting problems in energy consumption. Several popular statistical models for predicting energy consumption in buildings include autoregressive (AR) models such as AR, Autoregressive Integrated Moving Average (ARIMA), and variants of ARIMA model named Seasonal Autoregressive Integrated Moving Average (SARIMA). Other statistical regression algorithms are linear regression and multilinear regression, Bayesian regression, ordinary least square regression, and case-based reasoning.

The article "Deep Learning Neural Network Prediction System Enhanced with Best Window Size in Sliding Window Algorithm for Predicting Domestic Power Consumption in a Residential Building" was published in 2022. Journal: Comput Intell Neurosci.

AR model works on the fundamental of analyzing the statistical properties of energy-related time-series data. In other words, AR models predict future energy consumption only by considering the recent past and area data at a specific time. The implementation of these AR models was relatively simple and worked upon the theory of only looking back into the past data of dependent or target variables, but at the same time, these models have shown significant limitations, such that the forecasting horizon is limited to the short term only and cannot determine complex and nonlinear data patterns, which limit their application scope and accuracy [25–28]. However, researchers introduced several enhancements to overcome basic autoregressive models issues such as SARIMA models, Autoregressive Integrated Moving Average with Explanatory Variable (ARIMAX) models, and Seasonal Autoregressive Integrated Moving Average with Explanatory Variable (SARIMAX), but these improved versions of AR models are still facing some limitations accounting for not capturing nonlinear relationship within building energy-related time-series data, which highly affects the forecasting performance. In addition to these technical improvements, many researchers came up with the idea of hybrid models to tackle the above issues, such as ARIMA and Artificial Neural Network (ANN), ARIMA, and evolutionary models and collaboration with other machine learning algorithms [29–32].

On the other hand, statistical regression algorithms work on modeling the relationship between predictor and target variables. Various researchers predicted energy consumption in buildings by using linear regression [33–35], multiple regression [36, 37], and Bayesian regression [38]. Regression models suffer from multicollinearity problems that arise due to the relationship among independent variables used in prediction. Additionally, it is difficult to determine the explanatory variables, and we are still facing difficulty in dealing with the nonlinear problems.

#### 1.1.2. Traditional Machine Learning Modeling

Machine learning modeling acts as a black box and tries to learn the relationship that exists among input features and targets based on the provided data, such as energy performance. Several machine learning algorithms have been studied by researchers in buildings for estimating the energy consumption, energy demand, and their related performance criteria for different circumstances. Numerous techniques are widely used to analyze energy consumption prediction problems in various types of buildings, that is, commercial, residential, or industrial sectors.

The article "Deep Learning Neural Network Prediction System Enhanced with Best Window Size in Sliding Window Algorithm for Predicting Domestic Power Consumption in a Residential Building" was published in 2022. Journal: Comput Intell Neurosci.

Being a highly adaptable and flexible approach, ANN solved numerous prediction problems with respect to energy consumption [39–42], and nearly all the related works revealed that ANN outperforms real-time problems and identifies the nonlinear relations between input and output but at the same time deals with the several issues like overfitting problems when additional energy feature is introduced and local minima problems.

Besides that, support vector machines (SVM) are another efficient and widely popular modeling approach for solving nonlinear problems accounting for efficient energy management in buildings by forecasting energy consumption which covers [43–48]. These learning algorithms maintain a balance between nonlinearity and prediction accuracy. Though users find difficulty in identifying the kernel functions, an optimal hyperparameter will produce the optimal accurate prediction model. Users need to do a lot of rigorous work on the dataset properties and their own experience to deal with such issues.

There are other learning modeling employed black-box approaches used for different objectives such as detection and diagnosis of faults and forecasting energy consumption at different horizons with respect to buildings, with the focus of performance improvement covering ensemble models and improved hybrid models [49, 50].

Kim and Cho [16] predicted residential energy using a hybrid approach of deep learning, which uses a sliding window algorithm with fixed window size. The window size also affects the model performance. Besides that, model needs hyperparameter optimization as these parameters have a great impact on forecasting and model accuracy.

### 1.2. Contribution

The main contributions of this paper are as follows:

  This work proposes a Deep Learning Neural Networks prediction system enhanced with the best window size in sliding window algorithm for stably predicting domestic energy consumption in a residential building on 4.5 years of energy dataset
  The proposed deep learning models are tuned to achieve high performance based on various hyperparameters
  This study performs an extensive experimental evaluation of different variations of deep learning models and records the best RMSE value compared against the previous studies on the benchmark datasets
  This work also focuses on analyzing the variables of interest that construct the energy consumption data followed by various model fitting functions for a precise explanation of the electric consumption dataset

The structure of the paper is organized as follows: Section 2 provides a brief introduction to deep learning recurrent neural network theory.  Section 3 applies establishing deep recurrent neural network prediction models for domestic energy consumption in an actual residential house and analyzing various household appliances variables affecting the energy consumption forecasting, and performance measures and modification of hyperparameter for tuning the model performance will also be discussed in this section. In Section 4, the conclusions are presented.

The article "Deep Learning Neural Network Prediction System Enhanced with Best Window Size in Sliding Window Algorithm for Predicting Domestic Power Consumption in a Residential Building" was published in 2022. Journal: Comput Intell Neurosci.

## 2. Introduction to Deep Learning Recurrent Neural Network Theory

A specialized subset of machine learning is coined as “deep learning,” which [51–58] overcomes the accuracy issues [59]. Deep learning architectures are composed of nonlinear computation at multiple levels, such as neural nets performed by many hidden layers [60] with more abstraction and complexity. The key feature of deep learning architectures is automated feature extraction and data scaling with improved high performance [61]. Several artificial intelligence applications are widely relying upon the foundation of Deep Neural Networks. It includes robotics, IoT sensor data, image, speech recognition, and many other breakthrough domains that have exploded, which use Deep Neural Networks [62–66].

In this paper, the effectiveness of deep learning methods is explored by executing domestic level forecasting in a residential building. The proposed methodology uses CNN and LSTM techniques. The proposed work introduces an LSTM and CNN model with an enhanced sliding window algorithm. Both deep learning techniques are established on a benchmark electricity consumption dataset for an individual residential building with daily time resolutions.

### 2.1. LSTM for Time Series

Principally, neural networks for time-series forecasting are commonly categorized in two variants, namely, (i) feedforward neural networks and (ii) deep learning recurrent neural networks. Feedforward neural networks only process spatial information and skip temporal information, whereas deep learning recurrent neural networks are capable of handling both sequential and temporal information as it is composed of fully connected neurons having look back features even on a large-scale dataset. Regardless of these benefits, the typical recurrent neural networks (RNN) deteriorate due to vanishing gradient issues while handling the long-term dependencies [67].

The article "Deep Learning Neural Network Prediction System Enhanced with Best Window Size in Sliding Window Algorithm for Predicting Domestic Power Consumption in a Residential Building" was published in 2022. Journal: Comput Intell Neurosci.

Hochreiter and Schmidhuber [68] proposed a new advancement based on connected subnets to overcome the RNN shortcoming known as Long Short-Term Memory. LSTM has the ability to remember observations at arbitrary time lags. Now, the question is what makes LSTM remember? In conventional RNN, each cell receives two inputs, output from the previous hidden state and values at the “t” time. Apart from a hidden state, no past information exists to remember by the RNN. RNN cell representation is shown in Figure 1. The fundamental computations are provided in (1) and (2).

(1) $$\begin{array}{c} h^{t}=\sigma \left[W_{x}^{h}+x^{t}+W_{h}^{h}*h^{t-1}+b^{h}\right], \end{array}$$

(2) $$\begin{array}{c} Z^{t}=\sigma \left[W_{Z}^{h}*h^{t}+b^{Z}\right], \end{array}$$

where *σ* defines activation function, *W*_*x*_^*h*^, *W*_*h*_^*h*^, and *W*_*Z*_^*h*^ represent weight matrices of input, hidden, and output layer, and *b*^*h*^ and *b*^*Z*^ are bias at hidden and output layer, respectively.

A recurrently connected memory block uses memory cells with self-connections in addition to three multiplicative gates, namely, input gate (*i*_*t*_), input modulation gate (ć_*t*_), forgot gate (*f*_*t*_), and output gate (*O*_*t*_) in the hidden layer, enabling the model to store temporal state and to control the information flow in the network as directed by the associated activation function (ReLU, sigmoid, and tanh), thereby alleviating the vanishing of gradient problem. However, each gate plays a significant role.

  Input gate is responsible for writing operations
  Input modulation gate is responsible for the creation of a new cell value vector
  Forgot gate, also known as remember vector, is responsible for taking the decision of which information is to be kept or which is to be forgotten
  Output gate performs reading operations and decides which memory cell value passes to the next hidden state

Figure 2 shows the internal structure of LSTM. LSTM cell takes two inputs at “t” timestamp: (i) input at *t*(*X*_*t*_) and (ii) (*h*_*t*−1_) previous timestamps used to obtain the outcome. The working of each gate governs through a set of mathematical equations as presented in equations (3) to (7).

Cell state equation is as follows:

(3) $$\begin{array}{c} C_{t}=f_{t}*C_{t-1}+i_{t}*{\text{ć}}_{t}. \end{array}$$

Input gate equation is as follows:

(4) $$\begin{array}{c} i_{t}=\sigma \left(W_{i}*\left[h_{t-1},x_{t}\right]+b_{i}\right). \end{array}$$

Input modulation gate equation is as follows:

(5) $$\begin{array}{c} {\text{ć}}_{t}=\text{Relu}\left(W_{\text{ć}}*\left[h_{t-1},x_{t}\right]+b_{\text{ć}}\right). \end{array}$$

Forgot gate equation is as follows:

(6) $$\begin{array}{c} f_{t}=\sigma \left(W_{f}*\left[h_{t-1},x_{t}\right]+b_{f}\right). \end{array}$$

Output gate equation is as follows:

(7) $$\begin{array}{c} O_{t}=\sigma \left(W_{o}*\left[h_{t-1},x_{t}\right]+b_{o}\right), \end{array}$$

where *W*_*i*_,  *W*_ć _*W*_*f*_*W*_*o*_ define the weight matrices for input and recurrent layer and *b*_*i*_,  *b*_ć_, *b*_*f*_, *b*_*o*_ are the input and recurrent bias, respectively. Finally, the hidden state equation is defined for the output (*h*_*t*_) in equation (8), respectively.

The article "Deep Learning Neural Network Prediction System Enhanced with Best Window Size in Sliding Window Algorithm for Predicting Domestic Power Consumption in a Residential Building" was published in 2022. Journal: Comput Intell Neurosci.

Hidden state equation is as follows:

(8) $$\begin{array}{c} h_{t}=O_{t}*\text{Relu}\left({\text{ć}}_{t}\right). \end{array}$$

However, during the training process, the initial parameter values, that is, weights and bias of the LSTM, are generated arbitrarily. In general, weights and bias of the neuron in the LSTM layers can be updated through the standard gradient descent method employed by the backpropagation algorithm, but the performance of gradient descent highly depends upon the selection of optimal hyperparameters, which improves the accuracy of time-series problems.

### 2.2. CNN for Time Series

In general, there are a number of methodologies that perform analysis and prediction out of time-series data. However, these methodologies usually follow at least a two-step process: first, perform feature engineering and use some statistical algorithms or models to transform the time series as a vector of features; second, perform classification or regression tasks using various statistical or machine learning algorithms. On the other hand, CNN can be viewed as one frame architecture that incorporates the automatic extraction of features and modeling the time-series data. In this work, multivariate time-series data consists of “n” length and “k” width, where length defines time step count and width represents the total number of features. The CNN architecture viewed the input sequence as an image of “n” pixels and each pixel with “k” channels.

Unlike LSTM, CNN uses the current window and does not consider past information. The CNN consists of three layers, namely, input layer, multiple hidden layers, and output layer. The input layer receives extracted features as input, the output layer generates the prediction, and the hidden layer is further composed of three layers (convolution layer, ReLU layer, and pooling layer) and an activation function. Each sublayer of the hidden layer has a significant role in the prediction process: (i) Convolution layer uses convolution operation to the input sequence where convolution operation emulates the neurons' response, then processes the time-series data, and passes the outcome to the successor layer. (ii) ReLU layer is an activation function. (iii) Pooling layer is responsible for parameter reduction by reducing the space size for representation and thereby results in a reduction in computational cost. Equation (9) governs the *L*th convolution layer outcome, and equation (10) provides the working of the pooling layer.

(9) $$\begin{array}{c} y_{ij}=\sigma \left[\left(\overset{M}{\underset{m=1}{\sum }}W_{m,j}^{l}*X_{i+m-1,j}^{0}\right)+b_{j}^{l}\right]. \end{array}$$

(10) $$\begin{array}{c} P_{ij}^{l}=\frac{\text{Pooling Type}}{r\in R}\;\left(y_{i*T+r,j}^{l-1}\right), \end{array}$$

where *y*_*ij*_ is the output vector, *b*_*j*_ defines the bias, *W*_*m*,*j*_ defines the weight metrics, *m* defines the filter index value, *σ* is the activation function, *T* is the strides, *R* is the pooling size (must be less than the size of input), and pooling type defines which pooling function is used out of three: maximum, average, and sum, respectively. However, this work applies the “max” pooling type for parameter reduction.

The article "Deep Learning Neural Network Prediction System Enhanced with Best Window Size in Sliding Window Algorithm for Predicting Domestic Power Consumption in a Residential Building" was published in 2022. Journal: Comput Intell Neurosci.

Consequently, CNN transforms the given input sequence layer by layer. However, gradient descent will be used to train the weights and biases of the neurons in the convolution layer or fully connected layer so that the prediction scores computed by the CNN remain consistent with the training set.

### 2.3. Sliding Window Algorithm and Window Size

Sliding window algorithm is used to construct samples with one step size where each sliding window includes previous time steps as an input, and it aims to predict the upcoming time step. Consider the input vector *X*_*n*_ where subscript *n* is the number of normalized 7-day units to be taken per window. The sliding window algorithm is able enough to handle multivariate datasets as an input to the model and perform data smoothing of the original data by reducing the model time complexity. In the sliding window algorithm, the window size is quite responsible for deciding the number of time steps that need to be considered in the past and obtaining the optimal model as the model will learn the energy data that is preprocessed for every defined fixed window length. Consequently, the static window size may limit the temporal modeling in the deep learning neural networks as the data defined by the window size are only being modeled and are inappropriate to handle long-term dependencies in the time-series data.

To the best of our knowledge, most of the researchers used fixed or static window size in the sliding window algorithm. By selecting the proper size of a sliding window, the model efficiency can also be improved. Hence, this work is finding the best N window size in order to yield the best model with the least Root Mean Square Error. To accomplish this objective, an independent function is created, which takes a minimum value and maximum value as the parameters in order to observe the best window length for “N” previous time steps for prediction and run the deep prediction models several times to process the time series in each window using sliding window approach. For every “N” value, the window receives the input data from the beginning, and the time series is encoded into the vectors at the end of each window. Later, the obtained feature vectors are fed into the deep learning prediction models (i.e., LSTM and CNN) to estimate the prediction error with its respective training labels. In summary, Algorithm 1 presents the pseudocode for the deep prediction models with an enhanced sliding window algorithm.

The article "Deep Learning Neural Network Prediction System Enhanced with Best Window Size in Sliding Window Algorithm for Predicting Domestic Power Consumption in a Residential Building" was published in 2022. Journal: Comput Intell Neurosci.

### 2.4. Mathematical Formulation for Domestic Energy Consumption

In this work, predicting a domestic energy consumption problem has a multivariable time-series dataset with “N” distinct attributes, which include electrical measuring parameters and sensors deployed at different sections of residential buildings. At each time step “*t*,” electric energy consumed by the household appliances is recorded by the sensors attached to the submetering system and can be provided in the form of (11).

(11) $$\begin{array}{c} X_{t}=\left(X_{t}^{1},X_{t}^{2},X_{t}^{3},\;\ldots ,X_{t}^{n}\right), \end{array}$$

where *X*_*t*_^*n*^ signifies the total number of variables constitute energy consumption data at the “*t*” time step. Now, let us consider window size for input as this work includes a sliding window approach as follows:

(12) $$\begin{array}{c} WS_{k}^{l}=\left(X_{k},X_{k+1},X_{k+2},\ldots \ldots \ldots ,X_{k+l-1}\right), \end{array}$$

where *l* indicates the time-series length and training dataset with its labels represented as*l*_*i*_=*X*_*k*+*l*_. Therefore, models need to learn function “*f*,” which provide the mapping of window onto its respective training label and can be designed by (13).

(13) $$\begin{array}{c} l_{i}=\alpha \left(WS_{k}^{l}\right). \end{array}$$

So that, given energy consumption prediction problem can be transformed into supervised learning problem and uses Root Mean Square Error for prediction error. Hence, the prediction formal derivation is shown in (14).

(14) $$\begin{array}{c} {\text{Model}}_{\Omega }\min\frac{1}{2}\overset{N}{\underset{i=1}{\sum }}{\left(l_{i}-\alpha \left(WS_{k}^{l}\right)\right)}^{2}, \end{array}$$

where Model_Ω_ is the set of parameters for the model “*α*” and *N* is training size. Model “*α*” is a deep learning model like LSTM and CNN.

The article "Deep Learning Neural Network Prediction System Enhanced with Best Window Size in Sliding Window Algorithm for Predicting Domestic Power Consumption in a Residential Building" was published in 2022. Journal: Comput Intell Neurosci.

## 3. Establishing Deep Recurrent Neural Network Prediction Model for Domestic Energy Consumption

In this section, detailed explanations on the proposed deep learning recurrent neural network prediction system enhanced with an improved sliding window algorithm for accurate energy consumption forecasting will be provided.

### 3.1. Basic Electrical Energy Consumption of Residential Building Dataset Information and Data Preprocessing

In this study, the electric power consumption dataset was collected from the UCI machine learning repository [69]. The dataset contains the readings collected from the monitored house, situated in the city of Sceaux near Paris in France. This multivariate dataset is composed of recorded observations covering the period of 4 years from December 2006 to November 2010. During preprocessing, a total of 1.25% of the rows contain missing values that were imputed with the median. Also, redundant records are tried to be removed so that they will not cause the learning model to be biased towards the more frequent records during the training process[70].

Different electrical measures and submetering information of interest that construct the energy consumption data of residential buildings are presented in Table 2. The active power is the actual energy consumed, and the unutilized energy in the power line is referred to as reactive power. Besides active power, the dataset contains a distribution of real power via the main circuit in different areas of the home, that is, kitchen, washing area, and temperature control systems via sensory submetering systems, whereas voltage represents the average voltage supplied and global intensity refers to the average current intensity.

The major electrical energy consumption of a residential building can be divided into three categories: cookhouse consumption, lighting and utility room consumption, and heating and cooling system power consumption, as shown in Figure 3. From Figure 3, it can be observed that the energy used by the cookhouse and utility room along with lighting accounts for less impact on global power consumption. On the other hand, energy consumed by heating and cooling system accounts for a major portion of residential's electrical energy consumption. The equipment of the cookware house includes microwave, oven, and dishwasher that are connected to submeter 1, utility area includes lights, washing machine, drier, and refrigerator, which is connected to submeter 2, and heating and cooling units account for the water heater and air conditioner of the house concerned with the submetering 3.

The results of various model fitting functions are summarized for a precise explanation of the electric consumption dataset, as mentioned in Table 3. These fitting functions will help in estimating and understanding the distributional properties for different energy variables that are conditional on other variables and summarize the relationship among variables.

The article "Deep Learning Neural Network Prediction System Enhanced with Best Window Size in Sliding Window Algorithm for Predicting Domestic Power Consumption in a Residential Building" was published in 2022. Journal: Comput Intell Neurosci.

### 3.2. Applying LSTM and CNN Deep Learning Model

The proposed deep learning recurrent neural network protection system was implemented on the Anaconda Navigator using Python version 3.7 on an Intel Core i5 1.60 GHz processor with 8 GB ram on Windows 10 operating system. The whole experimental setup is divided into 3 steps, namely, (i) data preprocessing, (ii) data partition into training and testing dataset, and (iii) modification of hyperparameters.

#### 3.2.1. Data Preprocessing

A preliminary and inescapable phase in forecasting applications is used to reshape the obtained domestic electric power consumption dataset, from Section 3.1, into a proper format that can be fed into the learning model and aid in the convergence of the learning model. In this work, the z-score normalization technique was applied to the input features, thereby providing data transformation in such a way where the mean value equals zero and the standard deviation is 1 for the transformed data in order to prevent inaccurate predictions because of the presence of high-frequency components in energy consumption dataset. The mathematical formulation for z-score data transformation is shown in (15).

(15) $$\begin{array}{c} t_{i}=\frac{\left(t_{i}-\bar{t_{i}}\right)}{S_{i}};\;\forall \;i=\left(1,2,3,\ldots ,n\right), \end{array}$$

where $\bar{t_{i}}$ is the mean value of data samples, *S*_*i*_ defines the standard deviation of data samples, and *n* is the total number of data samples in the dataset. A significant highlight to be noted here is that prediction errors are recorded in their original scale in terms of various performance metrics, as discussed in Section 3.3.

#### 3.2.2. Data Partition

In the data partition step, the considered domestic energy consumption dataset is partitioned in order to generate training and testing data samples to reduce the learning model complexity and thereby optimize the accuracy. The dataset consists of 2075259 observations. For experiment, original energy data sampled at 1-minute granularity was later downsampled at the daily interval for meaningful analytics. Further, the sliding window approach was used for the short-term prediction of energy demand for a day. Initially, the sliding window of sequence size of seven points per window was considered, which is equivalent to 7 days in the past, in order to forecast the next point that is 24 hours or a day in the future.

The article "Deep Learning Neural Network Prediction System Enhanced with Best Window Size in Sliding Window Algorithm for Predicting Domestic Power Consumption in a Residential Building" was published in 2022. Journal: Comput Intell Neurosci.

Further to study the impact of window size on prediction error, sliding window approach enhanced with window size function which takes several ranges and tries to obtain the best N window size means the total number of days in the past that yields an optimal model with minimal prediction error as shown and discussed in Section 3.4. The training data samples for short-term prediction consist of energy consumption of a residential building for the period of three years using the aforementioned window size of 7 data points, and the rest of the one year of the energy dataset is held out purely for testing purpose.

#### 3.2.3. Modification of Hyperparameter

In general, hyperparameter is the model property governing the training process [70]. Hyperparameter covers two types of variables: one determines the model structure, and the other determines how the model is trained. Optimizing the hyperparameter has a significant impact on the performance of the model.

In this work, optimizer, activation function, neuron count in each layer, number of LSTM layers, kernel size, and kernel number (in case of CNN) followed by early stopping and model checkpoint hyperparameters were tuned to check out how these affect the model performance. Besides that, the dropout technique was used to perform regularization to avoid overfitting and generalization errors.

### 3.3. Performance Measures

The statistical measures are assessed to determine which model is suitable to amplify the goodness of fit using the classical model or hybridization of the model. In our work, the following set of statistical measures are selected to evaluate the prediction performance of the deep learning recurrent neural network prediction system over three states of the art of residential energy consumption, namely, Mean Square Error (MSE), Root Mean Square Error (RMSE), and coefficient of determination (*R*^2^). The statistical metrics are defined through equations (16)–(18), respectively.

(16) $$\begin{array}{c} \text{MSE}=\frac{1}{N}\overset{N}{\underset{\begin{array}{c} i=1\\ \left(y,\hat{y}\right)\in \text{Test} \end{array}}{\sum }}{\left(y_{i}-{\hat{y}}_{i}\right)}^{2}. \end{array}$$

(17) $$\begin{array}{c} \text{RMSE}=\sqrt{\frac{1}{N}\overset{N}{\underset{\begin{array}{c} i=1\\ \left(y,\hat{y}\right)\in \text{Test} \end{array}}{\sum }}{\left(y_{i}-{\hat{y}}_{i}\right)}^{2}}. \end{array}$$

(18) $$\begin{array}{c} R^{2}=1-\frac{\sum_{i=1}^{N}{\left(y_{i}-y_{i}^{\text{pred}}\right)}^{2}}{\sum_{i=1}^{N}{\left(y_{i}-y^{\text{mean}}\right)}^{2}}, \end{array}$$

where at time step “*i*,” *y*_*i*_ is the observed energy consumption, ${\hat{y}}_{i}$ is the predicted energy consumption, and “*N*” is the data point count in the test dataset.

The article "Deep Learning Neural Network Prediction System Enhanced with Best Window Size in Sliding Window Algorithm for Predicting Domestic Power Consumption in a Residential Building" was published in 2022. Journal: Comput Intell Neurosci.

### 3.4. Results of Deep Learning Models for Prediction of Domestic Energy Consumption

In this section, various experimental results are discussed for all variations of models implemented using LSTM and CNN enhanced with a sliding window approach. Also, a comparative analysis was performed to demonstrate the performance of the proposed model over competitive benchmarks using a household electricity energy consumption dataset. The main focus of this work is to implement a robust residential electricity energy consumption prediction system with minimal prediction error and high accuracy. The proposed model integrates both deep learning models, that is, LSTM and CNN, with the improved version of the sliding window algorithm, which is capable of identifying the best *n* window size and predicting the short-term energy consumption in a residential building located in the city of France. The parameter setting of the deep learning recurrent neural network prediction system enhanced with a sliding window algorithm is provided in Table 4. The LSTM and CNN models were implemented with TensorFlow at the backend, and the scikit-learn package was used for the implementation of other approaches in Python programming language on the Keras framework.

#### 3.4.1. Performance Comparison of All Model Variations for LSTM and CNN Models

A primary strategy was to conduct the experiments to find out the optimal LSTM and CNN network structure, that is, to tune various hyperparameters, as discussed in Section 3.2.3, while training the model using TensorFlow for predicting the household electric energy consumption scenario.

Tables 5 and 6 provide the details of hyperparameter tuning to observe how they affect the performance of the prediction system for predicting domestic energy consumption scenarios in terms of Mean Square Error and Root Mean Square Error. The above tables show the LSTM architecture with “Adam” optimizer (activation function = “ReLU,” dropout = 0.2, recurrent dropout = 0.2, neuron count = (128, 64), and LSTM layer count = 2) performing optimally for short-term prediction and CNN architecture with “Adamax” optimizer (activation function = “ReLU,” kernel size = (1,3), (1,1), kernel number = 64, 128, strides = (1,1), pool size = (1,1), and pooling type = “max”) executing in an optimal manner for short-term prediction.  Figure 4 and Figure 5 present single household electric power consumption prediction results of proposed deep learning neural network prediction system for short-term scenario, that is, one day ahead prediction of global power consumption.

#### 3.4.2. Optimal Window Size

This work confirmed the impact of changes in window size on deep learning models. Figures 6 and 7 present the optimal N window size graph for both LSTM and CNN models. The window size function takes several values to identify the best size for the sliding window as the fixed-size window length may limit the temporal modeling and also affect the model performance by increasing the forecasting error. Hence, this study analyzed and evaluated the proposed deep learning prediction system to be robust in the matter of dynamic window size and then compared the RMSE for the respective window size.

The article "Deep Learning Neural Network Prediction System Enhanced with Best Window Size in Sliding Window Algorithm for Predicting Domestic Power Consumption in a Residential Building" was published in 2022. Journal: Comput Intell Neurosci.

From the above figures, it was clear that LSTM with an improved sliding window algorithm gives better prediction performance with a window size of 7, 12, and 14, which means that these are the days that can be considered in the past sequence to obtain the minimal forecasting error. On the other hand, CNN with an improved sliding window approach provided minimal prediction error with the window size for 4, 5, and 8, respectively.

#### 3.4.3. Comparative Analysis with Competitive Benchmark

Further, a comparative study of the proposed work is performed with contrast benchmark models that use the considered household electricity consumption data. The prediction performance of the contrast model for the test dataset for daily time resolution is summarized in Table 7. Kim and Cho [16] stably predicted the total power consumption for a residential house using a hybrid approach by combining CNN and LSTM and applied a sliding window algorithm that enables the hybrid model to learn the input data. They fixed the window size to predict the minutely household consumption, but for the rest of the time resolutions like hourly, daily, and weekly, window size remains unclear. Chujai et al. [25] analyzed the energy consumption based on autoregressive models, that is, ARIMA and ARMA, using a benchmark dataset. They figured out forecasting errors for fixed and random window sizes. By comparing the error metrics, this work confirmed that the proposed deep learning recurrent neural network prediction system with an improved sliding window algorithm outperforms the considered contrasting benchmarks and also figured out the optimal window size for which the model achieved a minimal prediction error.

## 4. Conclusion

In this research work, an establishment of a residential energy prediction system is presented using the deep learning recurrent neural network; that is, LSTM and CNN models are used with an improved sliding window-based approach to establish a robust and accurate prediction of energy consumption in a residential building. This work employs a new feature in the sliding window algorithm of finding the optimal *N* value for window size that is the sequence length of data points to be considered in the past. This improvement does not limit the temporal modeling and yields an optimal model with minimal forecasting error.

The article "Deep Learning Neural Network Prediction System Enhanced with Best Window Size in Sliding Window Algorithm for Predicting Domestic Power Consumption in a Residential Building" was published in 2022. Journal: Comput Intell Neurosci.

A case study on individual household electric power consumption data collected from a residential building located in France to predict the total active power consumption for a day with daily time resolution, a short-term scenario, was presented. In this course of the evaluation, the impact of hyperparameter tuning was analyzed for the short-term scenario. Furthermore, the proposed deep learning prediction model outperforms benchmark contrast models in terms of different quality metrics like MSE and RMSE.

Although the proposed approach shows better prediction results, in the modeling process, the potential challenges are observed, which also provide a future directive to this study, as follows:

  Automating the hypertuning using some evolutionary approach
  Introducing additional features such as building parameters and occupancy parameters
  Impact of different time resolutions on model performance

## Figures and Tables

**Figure 1:** RNN cell representation.

**Figure 2:** Long Short-Term Memory cell unit representation.

**Figure 3:** Structure of electrical energy consumption of residential buildings.

**Figure 4:** Regression lift chart showing original and prediction values of household energy consumption using the LSTM model.

**Figure 5:** Regression lift chart showing original and prediction values of household energy consumption using CNN model.

**Figure 6:** Best N window size graph for LSTM model.

**Figure 7:** Best N window size graph for CNN model.

**Algorithm 1:** Deep prediction models with enhanced sliding window algorithm.

**Table 1:** Summary of researches conducted on energy consumption in buildings.

Technique	Focus of work	Sector and case study	Performance metrics	Pub.
ARMA and ARIMA	Analysis of household electricity consumption	French residential building (energy consumption data)	Akaike Information Criterion (AIC); Root Mean Square Error (RMSE)	[25]

ARIMA	Forecast the future demand	Residential building (power consumption)	Mean Square Error (MSE)	[51]

ARIMAX and ANN	Predicted hourly building load based on periodicity and linearity	Office building; ITES load data (electricity consumption and cooling)	AIC; mean bias error (MBE)	[29]

Linear regression and multiple regression	Prediction performance is analyzed based on hourly and daily time resolution	Residential building; TxAIRE Research and Demonstration House (energy consumption, weather data)	RMSE	[33]

ANN	Predicted energy consumption at a daily time resolution	Hong Kong-based office building (weather, building design parameters, and day type)	Nash–Sutcliffe efficiency coefficient; coefficient of variation of the Root Mean Square Error	[39]

Linear regression, feedforward neural network (FFNN), SVM, least-squares SVM, and hierarchical mixture of experts: regression and FFNN and fuzzy c-means with FFNN	Predicting one hour ahead electric energy consumption and a short-term forecasting scenario	Residential buildings; Campbell Creek 3 homes dataset (electricity consumption)	Coefficient of Variance (CV), Mean Absolute Percentage Error (MAPE), and MBE	[40]

Random forest	Predicting average and peak energy consumption based on people dynamics	Residential building; telecommunication data (electric energy consumption)	Mean Absolute Error (MAE), MSE, RMSE, Relative Squared Error (RSE), Relative Absolute Error (RAE), and coefficient of determination (R2)	[52]

SVM	Energy consumption prediction based on weather and building operating parameters	Commercial building; 3-star hotel energy dataset (weather data, lighting data, elevator, and cooling system data)	MSE; R2	[53]

Multilayer perceptron, linear regression, random forest, and SVM	Analysis and prediction of IoT-based sensor data in a building using different machine learning techniques followed by a rigorous comparative study with other learning techniques	Two-storey building (weather, light and appliances energy consumption, and temporal information)	R2, MAPE, MAE, and RMSE	[54]

Fuzzy Bayesian	To predict long-term energy consumption based on an econometric methodology to improve reliability and accuracy	Chinese per capita electricity consumption (PEC) dataset (electricity dataset)	MAE, MAPE, and RMSE	[55]

Ensemble bagging trees	Energy use prediction at hourly granularity	Institutional building; Rinker hall data (climatic, occupancy and temporal data)	R2, RMSE, and MAPE	[56]

LSTM	Forecasting energy load with one min and one-hour time resolution	Residential building; single house data (power consumption)	RMSE	[57]

Conditional Restricted Boltzmann Machine (CRBM) and Factored Conditional Restricted Boltzmann Machine (FCRBM)	The energy consumption forecasting over different time horizons (short, medium and long term) and on different time resolutions	Residential building; household electric dataset (energy consumption)	RMSE, R, and *p*-value	[58]

CNN-LSTM with fixed window size	Prediction of electricity consumption for next hour	Residential building; (electricity consumption dataset)	MAE, MAPE, RMSE, and MSE	[16]

The article "Deep Learning Neural Network Prediction System Enhanced with Best Window Size in Sliding Window Algorithm for Predicting Domestic Power Consumption in a Residential Building" was published in 2022. Journal: Comput Intell Neurosci.

**Table 2:** Different electrical measures and submetering information of interest that construct the energy consumption data.

**Variables**	**Description**	**Measuring units**
**Global active power**	Total active power	Kilowatts
**Global reactive power**	Total reactive power	Kilowatts
**Voltage**	Average voltage	Volts
**Global intensity**	Average current intensity	Ampere
**Submetering 1**	Active energy corresponds to the kitchen	Watt-hours of active energy
**Submetering 2**	Active energy corresponds to the laundry	Watt-hours of active energy
**Submetering 3**	Active energy corresponds to the cooling and heating appliances	Watt-hours of active energy

**Table 3:** Various model fitting functions for a precise explanation of the electric consumption dataset.

Fitting function	Min	1st quantile	Median	Mean	3rd quantile	Max	Standard deviation
Global active power	0.076	0.308	0.602	1.092	1.528	11.122	1.055
Global reactive power	0.000	0.048	0.100	0.124	0.194	1.390	0.113
Voltage	223.2	239.0	241.0	240.8	242.9	254.2	3.239
Global intensity	0.200	1.400	2.600	4.628	6.400	48.400	4.435
Submetering 1	0.000	0.000	0.000	1.122	0.000	88.000	6.139
Submetering 2	0.000	0.000	0.000	1.299	1.000	80.000	5.794
Submetering 3	0.000	0.000	1.000	6.458	17.00	31.000	8.436

**Table 4:** Parameter setting of the proposed prediction system.

Parameters	Range
Learning rate	(0.01,0.001)
Decay	(1*e* − 6)
Momentum	(0.9)
Beta_1	(0.9)
Beta_2	(0.999)
Epsilon	(None)
Batch size	128
Epoch	100

**Table 5:** Evaluation of different variations of LSTM model with sliding window algorithm.

Optimizer	Neuron count and number of LSTM layers	Activation function	Estimated Root Mean Square Error (RMSE)
SGD	128, 128, 128	ReLU, ReLU, sigmoid	0.0722
**Adam**	**128, 64**	**ReLU, ReLU**	**0.0693**
Adam	128	ReLU	0.0764
Adam	32	ReLU	0.0877

**Table 6:** Comparison of various model variations implemented by CNN with sliding window algorithm.

Optimizer used	Kernel size and kernel number	Activation function and layers	Estimated Root Mean Square Error (RMSE)
Adagrad	(1,3), (1,1) and 64, 128	ReLU and ReLU	0.1330
Adamax	(1,3), (1,1) and 128, 264	ReLU and ReLU	0.1201
Adam	(1,3), (1,1) and 64, 128	ReLU and ReLU	0.1183
**Adamax**	**(1,3), (1,1) and 64, 128**	**ReLU and ReLU**	**0.0836**
Adamax	(1,3), (1,3) and 64, 128	ReLU and ReLU	0.1110

**Table 7:** Prediction performance of contrast model.

Method	Time resolution	MSE	RMSE	*R* ^2^
ARMA [25]	Daily	—	0.34	
CNN-LSTM [16]	Daily	0.1037	0.3221	
LSTM	Daily	0.0048	0.0693	0.9679
CNN	Daily	0.0069	0.0836	0.9622

## Data Availability

The multivariate time series energy data used to support the findings of this study are available from the corresponding author upon request.
